RETRACTED

# Combination use of core decompression for osteonecrosis of the femoral head: A systematic review and meta-analysis using Forest and Funnel Plots

**DOI:** 10.1155/2021/1284149

**Published:** 2021-12-06

**Authors:** Linghanqing Wang, XuRong Tian, Keda Li, Chunlei Liu

**Affiliations:** ^1^Liaoning University of Traditional Chinese Medicine, Shenyang, 110847 Liaoning, China; ^2^Affiliated Hospital of Chengde Medical College, Chengde, 067000 Hebei, China

## Abstract

**Objective:**

This study evaluated the efficacy and safety of CD combined with bone marrow stem cells in the treatment of femoral head necrosis by systematic review and meta-analysis. *Methodology.* PubMed, The Cochrane Library, Embase, CNKI, Google Scholar and MEDLINE, etc. databases were searched for clinical randomized controlled trials (RCTs) comparing core decompression combined with autologous bone marrow mesenchymal stem cells versus core decompression alone in the treatment of femoral head necrosis. The retrieval period is from the establishment of each database to May 20, 2021. After literature was extracted and literature quality was evaluated, meta-analysis was conducted by using RevMan5.3 software.

**Results:**

A total of 420 osteonecrosis of the femoral head 452 patients' data were collected from all studies. Compared with the core decompression alone group, the CD combined with bone marrow stem cell showed marked reduction in the Visual analog scale (VAS), enhanced Harris hip score (HHS) at 12 months and 24 months, slowed down the progression of the disease, decreased the number of hips conversed to total hip arthroplasty (THA) in the future.

**Conclusion:**

Core decompression therapy is a very effective and safe treatment process used for ONFH. Moreover, CD combined autologous bone marrow stem cell transplantation can improve the survival rate of the necrotic head, reduce hip pain and delay the disease progression, the rate of THA postoperatively.

## 1. Introduction

The osteonecrosis of the femoral head (ONFH) is an obstruction or injury caused by the blood supply to the femoral head, resulting in bone tissue death. Subsequently, the restoration of osteocyte and bone marrow components leads to structural changes and disintegration of the femoral head, resulting in joint pain and disease which hard to heal for the patient [1–3]. Treating early-stage ONFH is still difficult and is a complex condition in the orthopedic field. Core depression (CD) is one of the most commonly used methods for treating early ONFH. Core decompression can reduce the pressure in the femoral head medullary cavity, it can break the necrotic part, improve blood flow resistance and venous reflux, intensify the substitution of the fresh bone, avoids femoral necrosis aggravated thus hindering the process of bone necrosis [4, 5]. A large number of studies revealed that core depression incorporated with cytotherapy is comparatively a superior treatment to turn down the rate of breakdown of early and mid-term osteonecrosis of the femoral head [6].

RETRACTED

There are two types of medications for ONFH: (1) surgical, and (2) non-surgical [7]. The non-surgical method comprises confined weight-bearing, medications, and biophysical methods. These treatments assist patients in the premature stages of the sickness with refined hip function, relief from the joint pain, and the probable avoidance of the radiographic subchondral rupture [8, 9]. The hip surgical methods included core decompression (CD), vascularized and non-vascularized bone implants, total hip arthroplasty (THA) [10, 11].

Bone marrow mesenchymal stem cells, also known as bone marrow stromal stem cells, is a kind of cell subgroup from mesoderm isolated from bone marrow tissue, which is capable to form organs and tissues such as bone, cartilage, or muscle [12–14]. In addition to bone marrow, BMSCs can also be isolated from adipose tissue, synovial tissue, umbilical cord blood, and other sources. BMSCs are easy to be isolated and culture. In animal experiments, researchers often isolate and culture BMSCs by extracting the femur and shin bone marrow of rabbits or mice, and clinically, surgeons separate BMSCs by extracting bone marrow tissue from the ala ossis ilium. BMSCs can be multi-directional differentiation, in condition medium, BMSCs can differentiate into bone, cartilage, and lipids, and BMSCs also have secretion functions, such as it can secrete insulin-like growth factors (IGF 1), vascular endothelial growth factor (VEGF), interleukin 6 (IL-6), stromal cell-derived factor⁃1*α*(SDF⁃1*α*) [15–17].

Some studies have shown that CD combined with bone marrow stem cell transplantation is better than CD alone in the treatment of femoral head necrosis. And as far as clinical trials establish the supremacy of the combined use of bone marrow stem cells and core depression [18, 19]. However, there is still some debate about whether transplantation can increase CD effectiveness. Therefore, this paper includes all clinical randomized controlled trials on BMSC transplantation combined CD and single CD comparison to treat ONFH, and systematically evaluates the safety and efficacy of BMSCs transplantation combined CD treatment on ONFH by forest and funnel plots, in order to more convincing conclusion.

## 2. Material and Methods

### 2.1. Search strategy

PubMed, The Cochrane Library, Embase, CNKI, Google Scholar and MEDLINE, etc. were systematically searched. Meanwhile, relevant reviews and references of included essays were searched manually, and the time limit of retrieval was set up until May 20, 2021. Keywords used for the search were "stromal cells", "bone marrow stromal stem cells," "Mesenchymal Stem Cells [Mesh], "core decompression", "ONFH", "osteonecrosis of the femoral head", "femur necrosis", "osteonecrosis", "bone marrow stem cells" etc.

RETRACTED

### 2.2. Inclusion criteria

- Study design was limited to randomized controlled trials (RCTs) and retrospective comparative studies (RTCs).
- Only those studies were included where patients were diagnosed with osteonecrosis in the femoral head with ARCO stage I - III or FICAT I-III
- When the trials were compared against by two types of studies; where there was the utilization of bone marrow stem cells (BMSC) along with core decompression (CD) group which was compared against core decompression (CD) alone group. Outcomes of the studies were evaluated on basis of Harris hip scores (HHS) at 12, 24 months, Visual analog pain scale, necrotic area of the femoral head, conversion to total hip arthroplasty (THA).
- The published studies with follow-up time≥ 1 year
- Reported mean, standard deviation (SD), range, and the number of subjects in each treatment for continuous outcomes.
- All studies included were published in English or Chinese.

### 2.3. Exclusion criteria's

Studies were excluded when

- The data shared the same set of information or repeated studies were removed.
- The study did not mention any major outcome
- Patients had comorbidities or reported other joint-based diseases like rheumatoid arthritis.
- Prognostic factors were not analyzed.
- Low-quality literature reports
- Animal studies regarding the topic were not included
- Case reports, editorial letters, meeting abstracts, guidance, review studies, and editorial comments were not included

### 2.4. Data extraction

The data from all the trials were extracted by 2 investigators of the study independently by using a format with sample size, age, lead author, disease stages, publication year, intervention, etiological factors, diagnostic criteria, inclusion and exclusion criteria, outcomes, and follow-up time. Cross-check after the extraction of the data, if there is any dispute, through discussion between the two sides to resolve, and a third researcher will be invited if necessary to rule.

### 2.5. Statistical Analysis

Revman5.3 software was used for Meta-analysis of the extracted data. The heterogeneity test of the results was carried out first, and meta-analysis was carried out using a fixed-effect model when I^2^ < 50%, indicating homogeneity between the studies. When I^2^ ≥50% indicates that there is no homogeneity between studies, the random-effects model was adopted. Continue data was represented by mean difference (MD) and 95% confidence interval (CI). We used odds ratio (OR) and 95% confidence interval (CI) for dichotomous outcomes. 𝑃 value< 0.05 was deemed statistically significant. The results of the analysis were represented by forest plots, publication bias was analyzed using a funnel plot.

RETRACTED

## 3. Results

### 3.1. Search results

By searching the database systematically, 536 articles were initially detected, and the remaining 104 were excluded after the exclusion of duplicate articles. After the full-scale screening, 10 clinical randomized controlled trials were finally included. A flowchart of articles selection is shown in Figure 1.

### 3.2. General characteristic of the included studies

A total of 420 patients were included in this meta-analysis. There were 214 patients in the combined utilization of BMSCs and CD group, and 206 patients in the CD alone group. Ten clinical randomized controlled trials included 420 cases of osteonecrosis of the femoral head and 452 hips. There were eight articles staged according to ARCO diagnostic criteria, and two articles used FICAT diagnostic criteria. The sample size of the patients ranged from 8 to 50. Follow-up duration ranged from 12 to 60 months. The basic characteristics of the included articles are shown in Table 1. According to the Risk assessment tool for RCT bias in the Cochrane Systematic Evaluator's Manual 5.1.0, the included studies were generally of moderate quality. The risk of bias summary and risk of bias graph was presented in Figures 2 and 3, respectively

### 3.3. Results of the meta-analysis

#### 3.3.1. VAS Score

Five trials compared the scores of Visual analogue scale (VAS) in two groups of patients after surgery. There is no homogeneity between studies (I^2^ = 96%, P < 0. 00001). For meta-analysis using a random-effect model, the results in Figure 4. **s**howed that the VAS score for hip pain after surgery in the experimental group was lower than that of the control group[MD=-7.01, 95%CI (-12.08,-1.94)]. Obviously, combination therapy can alleviate the pain of patients more than CD alone.

#### 3.3.2. HHS at 12 months and 24 months

The forest plot for meta-analysis of Harris hip score (HHS) at 12 and 24 months was presented in Figure 5. Harris hip score was recorded in five studies. The overall results indicated that the Harris hip score in the combined utilization of BMSCs and CD group was higher than that of the CD alone group at 12 months [MD = 8.08, 95% CI (3.98,12.19), P=0.0004, I ^2^ =74%] and 24 months [MD = 7.62, 95% CI (1.57,13.68), P = 0.0006, I ^2^=73%].

RETRACTED

#### 3.3.3. Disease progression

The forest plot for meta-analysis of disease progression was presented in Figure 6. Six studies including 306 hips reported disease progression postoperatively by using ARCO/FICAT staging to assess. There was homogeneity among the studies (I^2^=2%, P=0.40), and a fixed-effect model was used for meta-analysis. The results showed that the incidence of femoral head collapse and joint degeneration in the combined utilization of BMSCs and CD group was lower than that in the CD alone group [OR=0.15, 95% CI (0.07,0.32), 𝑃 value<0.00001].

#### 3.3.4. The rate of THA

Five studies involving 234 hips reported the future rate of total hip arthroplasty postoperatively. Slight heterogeneity existed between the five studies (I^2^=0%, P=0.51, Figure 7). Thus, a fixed-effects model was used. There was a significant difference between the two groups [OR=0.27, 95% CI (0.11,0.70), 𝑃 value=0.007]. The results of the meta-analysis showed that the combination group tended to reduce the future rate of THA compared with CD alone in the treatment of ONFH.

### 3.4. Publish bias analysis

The ten studies included were RCTs research, according to strict quality evaluation, Figure 8 showed the funnel plot of each observation indicator, showed that most of the observation data index base was centered on the vertical line, left and right sides, scattered evenly, can form a pyramid-like dotted line range, no obvious separation phenomenon, no obvious bias. Some of the results were slightly biased may be related to the small sample size of the literature included.

## 4. Discussion

The etiology and pathogenesis of osteonecrosis of the femoral head are complex, and there are many theories and no definite conclusion, which is also the reason cause the variety of treatment methods and poor efficacy [27]. The current theories include lipid metabolism disorder theory, bone marrow mesenchymal stem cell differentiation function decline theory, intravascular coagulation theory, cell apoptosis theory, and other theories that are the result of multiple mechanisms [28, 29]. Core decompression (CD) by drilling into necrosis areas is one of the most widely used treatments for ONFH, which improves bone marrow edema and increases blood flow supply [30]. At the same time, the CD can promote the regeneration of capillaries and bone girder, effectively repair bone tissue, improve local functional limitations, reduce hip pain, effectively delay Total hip arthroplasty(THA). Nevertheless, the repair of femurs has not been completely solved [31]. Studies have shown that the content of femur-near-end bone marrow-filled stem cells in patients decreased, and the ability to differentiate bone cells decreased [32, 33]. The decrease in femoral necrosis bone repairability may be related to the reduction of bone marrow interstate charge stem cell content and activity [34]. Therefore, in recent years, the local supplement of autologous bone marrow mesenchymal stem cells with CD has become a new trend to solve the problem of necrotic femoral head repair. After injecting cultured bone-derived stem cells into the muscles of ischemic rats, Kinnaird et al. [35]. found that gene expression levels of cytokines associated with angiogenesis (eg. VEGF, FGF-2, IL-6, etc.) increased and promoted lateral circulation and limb function recovery. Lebouvier et al. [36] treated femoral head necrosis in pigs by injecting BMSCs and found that BMCSs could significantly improve MRI imaging and histopathological changes in the necrotic area. A follow-up study of patients treated with BMSCs for up to 5 years found that autologous BMSCS transplantation significantly alleviated pain and delayed disease progression in ONFH patients [37]. In the early time, Hernigou [34] and Gangji [38] used autologous bone marrow cells respectively to repair defects after removal of necrotic lesions of femoral head. Both have achieved good results.

RETRACTED

In this systematic review, a total of 338 patients' data collected from all studies was evaluated for the study which belonged to different groups of treatments. This meta-analysis found that combination therapy is more effective than CD alone therapy alone to reduce postoperative pain and markedly improve hip function, delay the progression of femoral head necrosis, decrease the rate of THA in the future. And in the process of bone marrow stem cell transplantation and follow-up, no serious complications have been reported, so it can be considered that the treatment of osteonecrosis of the femoral head is safe and effective.

The present meta-analysis has several limitations. Firstly, the overall quality range was not high in the literature, the sample size was small. Second, the follow-up period of the article was not the same, the amount of bone marrow cell transplant received by patients was not the same, and the size of core decompression was not the same, which may result in potential bias. Third, published in Chinese or English may lead to regional or language bias. In the absence of more research and larger samples, more high-quality trials, including large samples and longer follow-up times, are recommended.

## 5. Conclusion

Core decompression is a safe and effective treatment for ONFH. The combination use of core decompression with BMSCs was also found to be more effective cause it can improv the Harris hip score, slow down the progression of osteonecrosis, even can reverse the disease staging. So core decompression combined with bone marrow mesenchymal stem cell transplantation treatment works better than alone core decompression and is worth promoting in clinical.

RETRACTED

## Figures and Tables

**Figure 1:** Flowchart for Selection of studies for meta-analysis.

**Figure 2:** The risk of bias of randomized trials included in the meta-analysis.

**Figure 3:** Risk of bias summary review authors' judgments about each risk of bias item for each included study.

**Figure 4:** Forest plot of the Visual analogue scale (VAS) score of patient's hip joint pain.

**Figure 5:** Forest plot of the Harris hip score (HHS) of patient's hip joint function at 12 months and 24 months.

**Figure 6:** Forest plot of disease progression shown by ARCO/FICAT staging.

**Figure 7:** Forest plot of the rate of total hip arthroplasty (THA).

**Figure 8:** The funnel plot of each observation indicator postoperatively. Note: Figure A-D is VAS, HHS, Disease progression, the rate of THA.

**Table 1:** The characteristics of included 10 studies.

Author	Country	Age (y, E/C)	Cases (n, E/C)	Sample size (hips)	Disease stages	Intervention	Control (drill diameter)	Follow-up(months)
FuQiang2013 [20]	China	37.5/36.1	23/22	32/29	ARCO: I-III	CD + BMSCs	CD(3.0mm)	12
Gangji2011 [19]	Belgium	42.2/45.7	13/11	13/11	ARCO:I/II	CD + BMSCs	CD(3.0mm)	60
GuoXiaowei2008 [21]	China	42/42	10/10	12/12	FICAT:I-III	CD + BMSCs	CD(2.0mm)	12
Hauzeur2017 [22]	Belgium	48.0/49.7	19/19	19/19	ARCO:I-III	CD + BMSCs	CD(4.0mm)	24
Pepke2016 [13]	Germany	44.3/44.5	11/14	11/14	ARCO: I/II	CD + BMSCs	CD(2.0mm)	24
Rastogi2013 [23]	India	34.7/33	30/30	30/30	ARCO:I-III	CD + BMSCs	CD(3.00m)	24
Sen2012 [24]	India	NA	26/25	26/25	ARCO:I-II	CD + BMSCs	CD(4.0mm)	60
Tabatabaee2015 [25]	Iran	31/26.8	14/14	14/14	ARCO:I-III	CD + BMSCs	CD(2.7mm)	24
Zhao2012 [7]	China	32.7/33.8	50/43	53/44	ARCO:I-II	CD + BMSCs	CD(1.0mm)	60
ZhaoRiguang2016 [26]	China	30.5/35.3	18/18	18/18	FICAT:I-II	CD + BMSCs	CD(3.2mm)	24

Note. E: experiment group. C: control group. ARCO: Association Research Circulation Osseous. FICAT: CD: core decompression. BMSCs: bone marrow stem cells.

## Data Availability

All data included in this study are available upon request by contact with the corresponding author.

## Abbreviations

CD: Core decompression
ARCO: Association Research Circulation Osseous
BMSCs: Bone Marrow Stem Cells
VAS: Visual analog scale
HHS: Harris hip score
ONFH: Osteonecrosis of the femoral head
MSC: Mesenchymal stem cells
THA: Total hip arthroplasty
